# Multivariate Analysis on Development of Lung Adenocarcinoma Lesion from Solitary Pulmonary Nodule

**DOI:** 10.1155/2022/8330111

**Published:** 2022-05-24

**Authors:** Linxiang Yu, Bin Zhang, Haosheng Zou, Yi Shi, Liang Cheng, Ying Zhang, Haiwen Zhen

**Affiliations:** Cardio-Thoracic Surgery, Affiliated Hospital of Nanjing University of Chinese Medicine, 210029 Nanjing, Jiangsu Province, China

## Abstract

**Objective:**

To analyze multiple factors developing lung adenocarcinoma lesion from solitary pulmonary nodule (SPN).

**Methods:**

A total of 70 patients diagnosed with lung adenocarcinoma after finding SPN by chest CT and treated in our hospital (01, 2018–01, 2021) were selected as the malignant lesion group, and another 70 patients diagnosed with benign lesion after finding SPN by CT in the same period were included in the benign lesion group. All patients had complete medical records. With univariate analysis and multivariate logistic regression, the independent risk factors for developing lung adenocarcinoma lesions from SPN were analyzed.

**Results:**

By conducting univariate analysis of patients' general information (age, course of disease, BMI, nodule diameter, and gender), smoking status (smoking history and number of cigarettes smoked per year), medical history (family history of lung cancer, history of extrapulmonary malignant tumor, and history of autoimmune diseases), basic complications (hypertension and diabetes), and laboratory examinations (CEA, NSE, CYFRA21-1, SCC-Ag, and CA125), it was concluded that age, course of disease, nodule diameter, CEA positive, CYFRA21-1 positive, and CA125 positive were significantly different between the two groups (*P* < 0.05); the logistic regression results showed that high age, increased nodule diameter, and CYFRA21-1 positive were the independent risk factors developing lung adenocarcinoma from SPN (*P* < 0.05).

**Conclusion:**

In patients with SPN, higher age, longer course of disease, greater nodule diameter, and CYFRA21-1 positive imply increased risk for triggering lung adenocarcinoma lesion. Therefore, high attention should be paid in the clinic to such SPN patients for early diagnosis and treatment.

## 1. Introduction

According to the global cancer statistics in 2018, lung cancer has the highest incidence and mortality worldwide, and it also ranks at the top of the incidence and mortality in China [1–4]. Despite the continuously improved diagnosis and treatment of lung cancer, relevant clinical data show that the 5-year survival rate of lung cancer remains less than 10%, which is mainly due to the fact that a large proportion of lung cancer patients are in the middle to advanced stage when diagnosed and miss the optimal period for surgical treatment. For early lung cancer patients, the 5-year survival rate can exceed 90% and the 10-year survival rate is about 88% after surgical resection of the lesions [5–8]. Lung adenocarcinoma is the most common histological type of lung cancer, with slow progression and insidious initial symptoms. Such patients tend to be detected by chest CT findings of lung nodules during physical examination, and distant metastasis is easy to occur at the advanced stage, presenting extremely poor prognosis. Therefore, early detection is of great significance in improving the survival rate of patients with lung adenocarcinoma. Most of the pulmonary nodules detected are single, thus also called solitary pulmonary nodules (SPNs), the nature of which is mostly benign nodules such as tuberculoma and pulmonary hamartoma, and malignant nodules are relatively rare, mostly primary early lung cancer, with the most common pathological type being adenocarcinoma and the second common type being squamous cell carcinoma [9–12]. There is a general consensus in the medical community that lung cancer is the result of the interaction of multiple factors, and lung nodules and lung cancer are closely related. At present, there are many studies on the prediction models of benign and malignant SPNs, but the prediction criteria are not consistent. Currently, the judgment of pulmonary nodules in the clinic is mostly based on medical imaging and physician's assessment of the characteristics of the medical history, among which the latter accounts for the majority [8]. Based on this, patients' clinical characteristics were analyzed herein to predict the risk factors for developing lung adenocarcinoma from SPN, in the hope of providing reference in this regard.

## 2. Materials and Methods

### 2.1. Screening and Grouping of Cases

A total of 70 patients diagnosed with lung adenocarcinoma after finding SPN by chest CT and treated in our hospital (01, 2018–01, 2021) were selected as the malignant lesion group, and another 70 patients diagnosed with benign lesion after finding SPN by CT in the same period were included in the benign lesion group. The study met the World Medical Association Declaration of Helsinki (2013) [13].

### 2.2. Inclusion Criteria

(1) The patients were found to have SPN (diameter ≤3 cm) via chest CT examination, with no clinical manifestations; (2) the patients did not have a history of malignant tumor; (3) the patients were diagnosed after pathological examination, and those with primary early lung adenocarcinoma and benign lesions were screened out; (4) the patients did not have remote metastasis; (5) the patients and their family members understood the study and signed the informed consent.

### 2.3. Exclusion Criteria for Patients

(1) History of lung cancer, with a diameter of pulmonary nodule over 3 cm; (2) multiple pulmonary nodules; (3) complicated with other lung diseases such as pneumonia and atelectasis; (4) complicated with dysfunction of important organs; (5) complicated with pleural effusion or mediastinal lymphadenopathy.

### 2.4. Statistics of Pathological Types

In the malignant lesion group, there were 5 patients with adenocarcinoma in situ, 25 patients with microinvasive adenocarcinoma, and 40 patients with invasive adenocarcinoma; and in the benign lesion group, there were 18 patients with hamartoma, 28 patients with inflammatory pseudotumor, 22 patients with pulmonary tuberculoma, and 2 patients with sclerosing hemangioma. See Figure 1.

### 2.5. Statistical Processing

The between-group differences were calculated with the software SPSS22.0 and analyzed with multivariate logistic regression, the picture drawing software was GraphPad Prism 7 Figure 2 (GraphPad Software, San Diego, USA), the items included were enumeration data and measurement data, which were expressed by (n (%)) and ($\bar{\text{x}}$  ± *s*) and examined by the X^2^ test and *t*-test, respectively, and differences were considered statistically significant at *P* < 0.05.

## 3. Results

### 3.1. Univariate Analysis

According to the univariate analysis, patients' age, course of disease, nodule diameter, CEA positive, CYFRA21-1 positive, and CA125 positive were statistically different between the malignant lesion group and the benign lesion group (*P* < 0.05) (see Table 1).

### 3.2. Multivariate Logistic Regression Analysis

According to the logistic regression analysis, higher age, increased nodule diameter, and CYFRA21-1 positive were the independent risk factors for developing lung adenocarcinoma (see Table 2) lesion from SPN (*P* < 0.05) (see Table 3).

## 4. Discussion

With the wide promotion of physical examination for the entire population and CT, the detection rate of SPNs has gradually improved. However, due to a large number of false positives, determining the nature of SPNs, especially lung adenocarcinoma, is very crucial, which is beneficial to improve the early diagnosis rate of lung adenocarcinoma, and has an important significance for selecting treatment modalities and patient prognosis [14–17]. At present, imaging data are the main clinical basis for characterizing pulmonary nodules, thus its clinical diagnosis has some subjectivity and the rate of misdiagnosis is high. Further statistics of patients in this study found that patients with malignant lesions were all adenocarcinomas, and most benign lesions were inflammatory pseudotumors, followed by tuberculosis spheres, which met the statistical results of previous studies. Therefore, emphasis can only be placed on clinical treatment with a clear pathological type of patients, which is also an important reference data to improve the subjectivity of the clinical diagnosis. In addition, preoperative percutaneous lung biopsy and bronchoscopic biopsy are commonly applied to obtain the accurate pathological diagnosis results, but with limited technique, equipment, etc., and many lung nodules are small in size and located deviate from the bronchus, so the acquisition rate of pathological positivity is usually not high. Although the clinical evaluation of pulmonary nodules cannot be used as a clinical diagnostic criterion for the determination of their nature, it can provide a reference for the screening of benign and malignant lesions of pulmonary nodules and the subsequent treatment, and combining the evaluation results with imaging and other examinations for multidisciplinary analysis also benefits the improvement of the sensitivity and accuracy rate of clinical diagnosis [18–21]. The study was to explore the affecting factors for developing lung adenocarcinoma lesions from SPNs, presenting a higher clinical application value for predicting the development of early lung adenocarcinoma in SPN patients. By conducting univariate analysis of patients' general information (age, course of disease, BMI, nodule diameter, and gender), smoking status (smoking history and number of cigarettes smoked per year), medical history (family history of lung cancer, history of extrapulmonary malignant tumor, and history of autoimmune diseases), basic complications (hypertension and diabetes), and laboratory examinations (CEA, NSE, CYFRA21-1, SCC-Ag, and CA125), it was concluded that age, course of disease, nodule diameter, CEA positive, CYFRA21-1 positive, and CA125 positive were significantly different between the two groups (*P* < 0.05); and the logistic regression results showed that high age, increased nodule diameter, and CYFRA21-1 positive were the independent risk factors for developing lung adenocarcinoma from SPN (*P* < 0.05). Related studies [22, 23] confirmed that the risk of malignancy will be increased in SPN patients at an advanced age, and the prediction model by William H. Amundson [24] et al. showed that more than 50% of patients with pulmonary nodules over the age of 60 years were confirmed as malignant lesions, whereas only 3% of patients under the age of 40 years had malignancy. Moreover, many references mentioned that smoking is the most common risk factor for lung cancer, and its exposure intensity and duration are proportional to the risk of lesions. This study confirmed that smoking was not an independent risk factor for SPNs to develop lung adenocarcinoma lesions, and no current research shows that smoking history has a strong correlation with adenocarcinoma.

In this study, measurement of tumor markers was included in the clinical evaluation for patients, which mainly included CEA, NSE, CYFRA21-1, SCC-Ag, and CA125 that were highly related to benign or malignant SPNs, of which CEA, CYFRA21-1, and CA125 presented significant differences in the univariate analysis, and the results of multivariate logistic regression analysis concluded that CYFRA21-1 could be the independent risk factor for developing lung adenocarcinoma lesion from SPN, and that the elevated CYFRA21-1 level might reflect SPN progression. CYFRA21-1 is an acidic polypeptide mainly found in the epithelial cytoplasm of lung tumors, which, in particular, has high sensitivity and specificity for the diagnosis of lung squamous cell carcinoma. CEA is a broad-spectrum tumor marker that is elevated in numerous tumors; CA125 is a nonspecific tumor marker often used in the treatment and prognostic monitoring of patients with ovarian tumors. CEA and CA125 were significantly different in univariate analysis but not in multivariate analysis, which may be related to their low specificity, so the sample size still needs to be expanded for further exploration in subsequent related studies.

To sum up, in patients with SPN, higher age, longer course of disease, greater nodule diameter, and CYFRA21-1 positive imply an increased risk for triggering lung adenocarcinoma lesion. Therefore, high attention should be paid in the clinic to such SPN patients for early diagnosis and treatment so as to promote the clinical diagnosis rate of SPN and guide the subsequent treatment for the patients.

## Figures and Tables

**Figure 1:** Statistics of pathological types of the malignant lesion group.

**Figure 2:** Statistics of pathological types of the benign lesion group.

**Table 1:** Statistics of patients' clinical data of the two groups.

Observation indicator	Malignant lesion group	Benign lesion group	X^2^/*t*	*P* value
General data				
Age (years)	61.03 ± 9.47	55.18 ± 10.44	3.472	<0.001
Course of disease (months)	10.94 ± 8.79	8.32 ± 6.47	4.403	<0.001
BMI (kg/m^2^)	24.61 ± 3.55	24.58 ± 3.49	0.050	0.960
Nodule diameter (cm)	2.54 ± 0.42	2.03 ± 0.61	5.761	<0.001
Gender (male/female)	38/32	40/30	0.116	0.734
Smoking				
Number of cases with history of smoking	21 (30)	22 (31.43)	0.034	0.855
Number of cigarettes smoked per year			0.193	0.661
≥400	15 (21.43)	17 (24.29)		
<400	6 (8.57)	5 (7.14)		
Medical history				
Family history of lung cancer	1 (1.43)	2 (2.86)	0.341	0.559
History of extrapulmonary malignant tumor	3 (4.29)	1 (1.43)	1.029	0.310
History of autoimmune diseases	2 (2.86)	3 (4.29)	0.207	0.649
Basic complications				
Hypertension	15 (21.43)	17 (24.29)	0.162	0.687
Diabetes	14 (20)	15 (21.43)	0.044	0.835
Laboratory examinations				
CEA positive	28 (40)	11 (15.71)	10.272	0.001
NSE positive	13 (18.57)	14 (20)	0.046	0.830
CYFRA21-1 positive	14 (20)	3 (4.29)	8.101	0.004
SCC-Ag positive	16 (22.86)	8 (11.43)	3.218	0.073
CA125 positive	24 (34.29)	10 (14.29)	7.614	0.006

CEA: carcinoembryonic antigen, the normal reference value is < 2.5 ng/ml; NSE: neuron-specific enolase, the normal reference value is < 16.3 ng/mL; CYFRA21-1 is a cytokeratin-19 fragment that is soluble in serum, and the normal reference value is < 3.3 ng/ml; SCC-Ag: squamous cell carcinoma antigen, and the normal reference value is ≤ 1.5 ng/ml; CA125: cancer antigen 125, and the normal reference value is < 35 U/ml.

**Table 2:** Multivariate logistic regression analysis.

Affecting factor	B value	S.E	Wals	df	Sig.	EXP (B)	95% CI of EXP (B)
Age	0.053	0.022	5.968	1	0.015	1.055	1.011–1.101
Diameter	2.020	0.442	20.864	1	0.000	7.540	3.169–17.940
CYFRA21-1	−2.031	0.831	5.976	1	0.014	0.131	0.026–0.669

The B value refers to the regression coefficient, EXP (B) refers to the odds ratio, S.E. stands for standard error, Sig. represents the significance, the Wald test is used to examine the B values, indicating the chi-square value, and df means the degree of freedom.

**Table 3:** Variable assignments.

Affecting factor	Name of variable	Instruction of assignments
Group	Group	Malignant lesion group = 1, benign lesion group = 0
Age	Age	Years
Course of disease	Course	Months
Nodule diameter	Diameter	cm
Carcinoembryonic antigen	CEA	Positive = 1, negative = 0
Cytokeratin-19 fragment antigen 21–2	CYFRA21-1	Positive = 1, negative = 0
Cancer antigen 125	CA125	Positive = 1, negative = 0

## Data Availability

The data used to support the findings of this study are available on reasonable request from the corresponding author.
